The article "Botnet Attack Detection in IoT Using Machine Learning" was published in 2022. Journal: Comput Intell Neurosci.

# Botnet Attack Detection in IoT Using Machine Learning

**DOI:** 10.1155/2022/4515642

**Published:** 2022-10-04

**Authors:** Khalid Alissa, Tahir Alyas, Kashif Zafar, Qaiser Abbas, Nadia Tabassum, Shadman Sakib

**Affiliations:** ^1^Networks and Communications Department, College of Computer Science and Information Technology (CCSIT), Imam Abdulrahman Bin Faisal University (IAU), P.O. Box 1982, Dammam 31441, Saudi Arabia; ^2^Department of Computer Science, Lahore Garrison University, Lahore 54000, Pakistan; ^3^Faculty of Computer and Information Systems Islamic University Madinah, Madinah 42351, Saudi Arabia; ^4^Department of Computer Science, Virtual University of Pakistan, Lahore 54000, Pakistan; ^5^Department of Finance and Banking, Jahangirnagar University, Bangladesh

## Abstract

There are an increasing number of Internet of Things (IoT) devices connected to the network these days, and due to the advancement in technology, the security threads and cyberattacks, such as botnets, are emerging and evolving rapidly with high-risk attacks. These attacks disrupt IoT transition by disrupting networks and services for IoT devices. Many recent studies have proposed ML and DL techniques for detecting and classifying botnet attacks in the IoT environment. This study proposes machine learning methods for classifying binary classes. This purpose is served by using the publicly available dataset UNSW-NB15. This dataset resolved a class imbalance problem using the SMOTE-OverSampling technique. A complete machine learning pipeline was proposed, including exploratory data analysis, which provides detailed insights into the data, followed by preprocessing. During this process, the data passes through six fundamental steps. A decision tree, an XgBoost model, and a logistic regression model are proposed, trained, tested, and evaluated on the dataset. In addition to model accuracy, F1-score, recall, and precision are also considered. Based on all experiments, it is concluded that the decision tree outperformed with 94% test accuracy.

## 1. Introduction

The proliferation of the Internet of Things (IoT) devices has resulted in a steady rise in the volume of IoT-based assaults.. One of the most serious IoT risks is the IoT botnet attack, which tries to commit actual, effective, and profitable cybercrimes. IoT botnets are collections of Internet-connected IoT devices that have been infected with malware and are managed remotely by an attacker [1].

The Internet of Things (IoT) systems have significant challenges in offering techniques to detect security vulnerabilities and assaults due to the rapid growth of threats and diversity in attack tactics. As malware is executed, there have been an increasing number of improvements in machine learning/deep learning-based detection tools and techniques that use full-time series data. However, the need to employ full-time series data severely limits existing works' usefulness [2]. On the other hand, earlier identification would enable better IoT Botnet response proposals. As a result, it reduces the harm caused by possible assaults. The dynamic analysis method examines how malware interacts with its surroundings when it is being executed [3].

The article "Botnet Attack Detection in IoT Using Machine Learning" was published in 2022. Journal: Comput Intell Neurosci.

These data are extremely important for machine learning and deep learning models detecting malware. The representative approaches required continuous series data collection while the malware is running [4]. In this instance, the malware successfully carried out its goal of information system sabotage and fully exhibited its hostile nature. There are currently available detection techniques for such stages, thus if a DDoS assault performed by an IoT Botnet has already taken place, identifying the DDoS attack, and the IoT Botnet network by itself at this point is not too challenging [5].

The use of bot malware and botnets to support other harmful online activities (such as click fraud, distributed denial of service attacks, and spam and virus distribution). The IoT Botnet lifecycle includes a lengthy scan and propagation phase. If it is feasible to identify and isolate the bots before they launch an actual assault, such as a DDoS, the IoT Botnet detection solution will have a stronger impact [6]. Therefore, it is crucial and required to identify harmful actions of IoT Botnet network components as soon as possible. However, it might be difficult to identify botnets, especially peer-to-peer (P2P) botnets [7]. As a result, we provide a complex traffic reduction strategy in this study that is coupled with a reinforcement learning method. Unquestionably, one of the most fascinating divisions of AI is machine learning. It successfully completes the goal of learning from data with specific machine inputs. It is crucial to understand how ML operates and, consequently, how it might be applied in the future. Training data [8] are entered into the chosen algorithm to begin the machine learning process. The final ML algorithm is developed using the training data, which might be known or unknown data. The method is affected by the type of training data input, and that idea will be discussed in more details shortly [9].

The machine learning algorithm is fed fresh input data to see if it functions properly. Then, the prediction and outcomes are cross-checked [10]. The algorithm is repeatedly retrained if the prediction and results do no't line up until the data scientist achieves the desired result. As a result, the ML algorithm is able to continuously train on its own and produce the best solution, steadily improving in accuracy [11].

The article "Botnet Attack Detection in IoT Using Machine Learning" was published in 2022. Journal: Comput Intell Neurosci.

### 1.1. Types of Machine Learning

The study of machine learning encompasses a wide range of topics and draws inspiration from other domains, including artificial intelligence. The field is centered on learning or gaining abilities or knowledge through practical application. Usually, this entails pulling relevant concepts from the previously collected data. As a result, in the field of machine learning, you may come across a wide variety of learning, ranging from entire fields of study to particular methodologies. Different types of machine learning as shown in Figure 1.

Due to its complexity, machine learning has been separated into two main categories: supervised learning and unsupervised learning, and two ancillary categories: semi-supervised learning and reinforcement learning. Each one has a distinct goal and course of action that produces outcomes and uses different types of data. Supervised learning makes up over 70% of machine learning, whereas unsupervised learning is between 10% and 20%. Semi-supervised and reinforcement learning take up the remaining space.

## 2. Problem Statement

In distributed computing environments, remote access to services has become widespread due to the Internet. Nonetheless, the integrity of data transmission on the distributed computing platform is hindered by security concerns. Botnets are a prominent threat to Internet security, as are malicious codes. In addition to distributed denial of service (DDoS) attacks, click fraud, phishing, malware distribution, spam emails, and the illegitimate exchange of information or materials, botnets support a wide range of criminal activities. Therefore, developing a robust mechanism for detecting, analyzing, and removing botnets are imperative. At present, botnet detection techniques are reviewed in a variety of ways. However, studies of this type are limited in scopes and lack discussions about the newest botnet detection techniques. The aim of this study is to develop a state-of-the-art machine learning model for botnet detection, utilizing the latest emerging techniques, and analyzing current and past research trends. The study offers a thematic taxonomy for classifying botnet detection techniques and analyses such techniques' implications and critical elements.

## 3. Research Motivation

The field of cybersecurity is always a challenging task for researchers. As a result, cybercriminals constantly research new approaches to identify weaknesses and use them for nefarious and illegal purposes. Malware spreading technique is now growing with new and innovative manners. The malware is then used to carry out further attacks like data exfiltration and denial of service attacks utilizing or on compromised machines.

The article "Botnet Attack Detection in IoT Using Machine Learning" was published in 2022. Journal: Comput Intell Neurosci.

## 4. Significance of Our Study

Internet of Things (IoT) services and applications have significantly increased due to their functionality and ease of use. Companies have started to develop a variety of Internet of Things (IoT)-based products, ranging from modest personal gadgets like a smartwatch to an entire network of smart grid, smart mining, smart manufacturing, and autonomous driverless vehicles. The overwhelming quantity and ubiquitous presence have enticed potential hackers for data theft and cyberattacks. One of the most significant issues with the Internet of Things is security. This study's main objective is to suggest a novel machine learning algorithm-based model for detecting and thwarting botnet attacks on IoT networks.

## 5. Research Objectives

The objectives of this study are as follows:

1. To transform the raw data into machine learning format using data transformation and preprocessing techniques.
2. To develop the machine learning model which will be used to classify the botnet attacks.

## 6. Literature Review

The well-organized intrusion representations are used to analyze current and upcoming network outbreaks [12]. Several machine learning algorithms have been established. In this research, a UNSW-NB15 dataset was cast off before the standard KDD99 data set, which depicts current complex attacks and network traffic. An extreme gradient is one of many machine learning algorithms boosting (XGBoost), which delivers extremely efficient and precise data. A subset of the results was chosen. 23 of the 39 useable characteristics were achieved through information gain. Various classifiers such as neural network, multi-logistic regression, nonlinear svm, XGBoost, Naïve Bayes, and random forest are trained and evaluated. From all the XGBoost outperformed with 88% test accuracy, followed by random forest which reported 87.89% accuracy [13].

More experiments were conducted, and the researchers looked up a Deep Neural Network (DNN) for detecting IoT attacks. DNN's ability to correctly identify attacks has been tested on the most commonly used data sets, including KDD-Cup'99, NSL-KDD, and UNSW-NB15. The experimental results demonstrated the precision rate of the projected method using the DNN. It demonstrated that each data set's accuracy rate is greater than 90%. As accuracies reported on the KDD-Cup'99, NSL-KDD, and UNSW-NB15 datasets are 96.30%, 91.50%, and 99.20%, respectively [14].

Similarly, numerous other studies have been conducted in which experts adopt deep learning to detect intrusion. The research includes the deep learning models ANN, DNN, and RNN as an interruption detection system. The dataset UNSW-NB15 was established in diverse files and then categorized into binary classifications with deep learning models to measure abnormal patterns. In this study, the whole dataset was combined in a solo folder for models being tested more fairly than separately for a separate file. The dataset attack families were then used as new labels, resulting in a multi-classification labelled dataset. The improved dataset categorized deep learning performance into dual arrangement groups (Binary and Multi-Class). The deep learning models that we propose show the accuracy in multi-class classification was 99.59%, and the accuracy in binary classification was 99.26% [15]. The comparison between research shows the competence of DL and ML representations in the improved dataset using accuracy and loss.

The article "Botnet Attack Detection in IoT Using Machine Learning" was published in 2022. Journal: Comput Intell Neurosci.

The paper proposed and tested the IGRFRFE fusion collection technique on behalf of MLP incursion concealment systems on the UNSW-NB15 modern IDS set. IGRFRFE is made up of two feature reduction steps, one of which is IGRF recursive feature elimination with MLP and ensemble feature selection. The screen option collection technique was used to reduce the feature subset search space, which is a mixture of IG and RF Importance. Then, as a wrapper feature collection method, recursive feature elimination (RFE) was used to eliminate terminated features on the concentrated feature subsets. The effects indicate that the option measurement is concentrated from 42 to 23, while the MLP precision is upgraded from 82.25% to 84.24%. The outcomes on the UNSW-NB15 dataset authorize that the projected process can expand irregularity, and detection accuracy while dropping feature measurement [16].

ML methods can detect data based on prior experience and distinguish between normal and abnormal data. The CNN DL technique was established in research work conducted in 2021 to resolve the difficulties of identifying network intrusion. The CNN algorithm was accomplished using the UNSW NB15. In general, the data covers binary types for usual and attack data. The tentative results verified that the anticipated model accomplishes extreme detection accuracy of 93.5%, and also evaluation metrics were used to amount to the performance of the CNN algorithm [17].

According to the tentative results, the original KDD99 features are less effective than the KDD99 data set's simulated UNSW-NB15 features. However, when datasets are compared, the precision of the KDD99 dataset is higher than that of the UNSW-NB 15. The FAR of the KDD99 is lesser than that of the UNSWNB 15 dataset. However, the reported accuracy of the proposed model is 98.89% [18].

The article "Botnet Attack Detection in IoT Using Machine Learning" was published in 2022. Journal: Comput Intell Neurosci.

Recent improvements in machine learning consumed a preferred tool for various classification and analytical difficulties. The analysis provides information, investigates challenges, fundamental analyses of data in terms of security, and forecasts future opportunities for machine learning in networking. From all the proposed classifiers, the random forest outperformed with 86.99% accuracy while Ada boost performed the least with 83.67% test accuracy [19].

## 7. Solution Design and Implementation

### 7.1. Conceptual Description of the Solution

The methodology proposed for this research has strictly followed the classical machine learning pipeline. Following all steps, the data was passed to the proposed classifiers and evaluated. The flowchart of modelling can be illustrated in Figure 2.

Whenever a dataset project is undertaken, the first phase involves the collection of datasets. For this research, the well-known dataset known as UNSW-NB15 has been collected from Kaggle. The dataset was then passed through the exploratory data analysis (EDA) phase to perform the statistical analysis and get meaningful insights into dataset attributes [20].

The proposed methodology consists of feather extraction, traffic reduction, and a multi-layer network classifier to detect the botnet from the normal traffic. In the first phase, traffic is reduced by filtering the TCP control packet after the feather extraction. After extracting the features, the model is trained for botnet detection and legitimate traffic, as shown in Figure 3.

### 7.2. Dataset Description

In this research, the models are built and trained to classify the botnet attacks. For this purpose, a publicly available dataset known as UNSW-NB15 is collected from Kaggle [21]. The dataset is published by the IXIA Perfect Storm tool. The Australian Centre for Cyber Security (ACCS) is an authentic botnet classification dataset. The UNSW-NB 15 dataset was created by the IXIA PerfectStorm tool in the Cyber Range Lab of the Australian Centre for Cyber Security (ACCS) to generate a hybrid of real modern normal activities and recent synthetic attack behaviors [22].

This dataset has nine attacks labelled, such as Fuzzers, Analysis, Backdoors, DoS, Exploits, Generic, Reconnaissance, Shellcode, and Worms [23–25]. Using the tools Argus, and Bro-IDS, 12 algorithms have been developed to generate a total of 49 functions in class labels. These features are described in the UNSW-NB15_features, csv file. The total number of records is 2 million and 540,044 are stored in four CSV files UNSW-NB151 csv, UNSW-NB152 csv, UNSW-NB153 csv, and UNSW-NB154 csv. The name of the ground truth table is UNSW-NB15 GT csv and the name of the list of event files are UNSW-NB15LIST_EVENTS csv.

The article "Botnet Attack Detection in IoT Using Machine Learning" was published in 2022. Journal: Comput Intell Neurosci.

The partitions for this dataset are configured as training sets and test sets, namely UNSWNB15training-set csv and UNSWNB15testing-set csv, respectively. The training set has 175,341 records, and the test set has various types of attacks and regular 82,332 records.

The dataset has 45 attributes. Details of attributes are described in Table 1.

This is a binary class classification dataset as its label column has just two values (0 and 1). 1 represents that it is the attack record else 0 in the case of a normal record. In total, the dataset has 30 integers, 11 floats, and 4 categorical attributes.

The acute process of performing an initial investigation on data to discover patterns, spot noise, and outliers, to test a hypo study, and to check assumptions with the help of summary statistics and graphical representation is called exploratory data analysis and is commonly known as EDA. When analyzing a dataset, it is important to do both statistical and graphical analyses.

The visualization reveals that this is the binary class classification dataset as it has only 2 classes (0 and 1). Secondly, the dataset is highly imbalanced as the 0 class is almost half of 1. The count of class 1 and 0 is 164673 and 93000, respectively as shown in Figure 4. If this thing remains unhandled then the model will not be trained accurately, affecting the model performance and leading to the miss classification.

This is the frequency chart of the attack cat column, representing 10 different categories of attacks, out of which the normal is the highest and the worm's category has the minimum frequency as shown in Figure 5. Other categories are generic, exploits, fuzzers, DoS, surveillance, analysis, backdoor, and shellcode. The proto is an attribute which enlists all the transaction protocols. It has 10 unique values, including tcp, udp, ospf, gre protocols, and the percentage of each protocol is present. Tcp has the highest frequency, followed by udp where ipv6 occurred the most least.

Figure 6 and Figure 7 are illustrations of service and state protocol, respectively. The service attribute has 11 unique values, of which 7 attributes' frequency almost equals to zero, whereas the state attribute has 13 unique values, around which 5 attributes have a frequency which almost equals to zero. Skewness is a measure of asymmetry or distortion of symmetric distribution. It measures the deviation of the given distribution of a random variable from a symmetric distribution, such as normal distribution. A normal distribution is without any skewness, as it is symmetrical on both sides. Hence, a curve is regarded as skewed if it is shifted towards the right or the left. The skewness of all numerical features of this research is shown in Figure 8.

The article "Botnet Attack Detection in IoT Using Machine Learning" was published in 2022. Journal: Comput Intell Neurosci.

All the numerical attributes have normal skewness and most of them are either left or right skewed. Only the id column has normal distribution because it has all unique values.

Values range from 0 to 60. Most of the values are close to 0 and lesser than 20. ct_dst_ltm highly corr with ct_dst_sport_ltm ct_src_ltm corr with ct_src_dport_ltm ct_src_dport_ltm corr with ct_dst_sport_ltm.

Numerical feature with a small discrete set of values. Normal data has 0 as most of its values. Anomaly has most of its value 2. There are few attacks with a value 1 and very little nonattack with 1.

This feature has 55 unique values. Attack data has value 0 most of the time, but that is also way too little compared with nonattack data. Most of the nonattack data have value of 1 and very few 2,3,4, 19,21,23 but very few in number not visible in the graph a.

Figure 9 has a range up to 800,000. Normal data is distributed over a very wide range up to 200,000. For attack data, there is a huge peek close to 0, and distribution of values is very narrow, whereas the Dload feature has a high correlation with target feat, the 0.35 Feature has a huge range of values up to 1e8. We can visualize better in a log scale. Normal data are distributed all over, has values close to 0 and very large values; for attack data, all the values are very close to 0. IN log scale we can see that values are between 3 and 15.

Most of the values for nonattack data are 29. There are some 0 and very few 252, as shown in Figure 10. There are lots of 0 in attack data, no of 0 in attack is more than nonattack, and 252, which is also higher than nonattack. Boxplots are used to visualize the outliers/noise present in data. The most important attributes have been visualized using a boxplot.

These are the boxplots of attributes labels, is_sm_ips_ports, ct_src_ltm, response_body_len, swin, dttl and sttl as shown in Figure 11.

Figure 12 illustrates the attributes attack cat and no of events. The second and most important step of any machine learning project is dataset processing. Hence the dataset is in raw format and cleaned it, and transformed the data into the form acceptable by machine learning classifiers.

### 7.3. Data Pre-processing

The data mining technique used to convert raw data into valuable information for machines is known as preprocessing. The following steps have been performed in preprocessing. It is observed that the real-world data is often incomplete, is inconsistent, and contains a lot of errors.

The article "Botnet Attack Detection in IoT Using Machine Learning" was published in 2022. Journal: Comput Intell Neurosci.

As illustrated in Figure 13, datasets are preprocessed by using the given fundamental steps.

#### 7.3.1. Handle Null/Missing Values and Duplicate Data

Fortunately, the dataset has no null or missing values, as shown in Figure 14. Moreover, there is no redundant data too. Till this point, the dataset is clean, but *i* need further preprocessing such as label encoding and feature extraction.

### 7.4. Label Encoding

The dataset has four categorical columns that need encoding to feed into the model. To transform it into a numeric form, the label encoder is used.

Figure 15 and Figure 16 shows the before and after of encoding, and all the data has been transformed successfully.

### 7.5. Feature Engineering

One of the most crucial steps of preprocessing is a selection of features. There are many ways of feature selection. The most suitable features have been extracted and selected for this research using the correlation technique.

Three types of correlation exist between the features: neutral, positive, and negative.  Figure 17 illustrates the heap map of correlation that exists between the features. With 0.4 threshold the discarded features are ‘id', ‘sloss', ‘dloss', ‘dpkts', ‘dwin', ‘time', ‘ct_srv_dst', ‘ct_src_dport_ltm', ‘ct_dst_src_ltm'. These features negatively correlate with label and will affect the model negatively.

### 7.6. Balance Dataset

Imbalanced data typically refers to a problem with classification problems where the classes are not represented equally. Most classification data sets do not have an exactly equal number of instances in each class, but a slight difference often does not matter.

Specialized techniques which can be used to balance the dataset are

1. Under-sampling
2. Oversampling
3. SMOTE

In this research SMOTE oversampling has been used. SMOTE is a technique generally known as Synthetic Minority Oversampling Technique. This is a systematic algorithm used to generate synthetic samples. As the name implies, SMOTE is an oversampling method. Instead of making a copy, it works by making a synthetic sample from a subclass. The algorithm selects two or more similar instances (using a distance measure). It perturbs one instance with one attribute at a time, in random quantities within the range of differences from adjacent instances. After applying the SMOTE oversampling technique, the dataset is now balanced, and the final shape of the dataset is (329346,37) instead of (257673,36). Now the dataset is cleaned, transformed, and balanced. It is ready to train a machine learning model.

## 8. Result and Analysis

Three machine learning classifiers, Decision Tree, XgBoost, and Logistic Regression, are trained, tested, evaluated, and compared in this dataset. The comparative analysis is also performed for both unbalanced and balanced datasets.

The article "Botnet Attack Detection in IoT Using Machine Learning" was published in 2022. Journal: Comput Intell Neurosci.

### 8.1. Decision Tree

Firstly, the dataset was split into train and test by using the train test split method. 80% was used for training, while 20% was used for testing. This model was trained for both balanced and unbalanced datasets, and the following results have been achieved in Table 2.

From Figure 18 and Figure 19 we can see that all the evaluation parameters (precision, recall, and f1-score) are 100, which indicates that there is a problem in learning. The model is only learning one class and miss classifying other.

These are the confusion matrix in which there is no true negative and false positive for an unbalanced dataset present in Figures 20 and 21.

### 8.2. XgBoost

XgBoost is a boosting classifier with 80% training and 20% testing. The model was trained for both balanced and unbalanced datasets, and the following results have been achieved as shown in Table 3.

From Figures 22 and 23 we can see that all the evaluation parameters (precision, recall, and f1-score) are 100, indicating a problem in learning, and the model is only learning the one class and miss classifying others.

Unlike the balanced dataset confusion matrix, there is no classification in the unbalanced dataset confusion matrix as shown in Figures 24 and 25.

### 8.3. Logistic Regression

Logistic regression is the regression technique used to classify binary data. In this 80% training and 20% testing split dataset has been passed to the model for training of both balanced and unbalanced dataset, and the following results have been achieved as shown in Table 4.

From Figures 26 & 27, we can see that all the evaluation parameters (precision, recall, and f1-score) are 100, indicating a problem in learning. The model is only learning one class and miss classifying others. The performance of logistic regression was not good compared to the decision tree and XgBoost.

From all the trained models, the decision tree outperformed with a slightly higher accuracy than the decision tree by predicting a few true positive values and logistic regression has the least performance.

These confusion matrix results are the same for the unbalanced dataset as there is no true negative and false positive present unlike the balanced dataset confusion matrix, there is no classification there, as shown in Figures 28 and 29.

The charts summarized all the results and experiments of this research. With a balanced dataset, the decision tree outperformed with 94% accuracy, as shown in Figures 30 and 31.

The article "Botnet Attack Detection in IoT Using Machine Learning" was published in 2022. Journal: Comput Intell Neurosci.

## 9. Conclusion

Cyber-attacks involving botnets are multi-stage attacks and primarily occur in IoT environments; they begin with scanning activity and conclude with distributed denial of service (DDoS). Most existing studies concern detecting botnet attacks after IoT devices become compromised and start performing DDoS attacks. Furthermore, most machine learning-based botnet detection models are limited to a specific dataset on which they are trained. Consequently, these solutions do not perform well on other datasets due to the diversity of attack patterns. In this work, UNSW-NB15, the most generalized dataset publicly available, is used. EDA (Exploratory Data Analysis) is the statistical analysis phase through which the whole dataset is analyzed.

The model will be able to be trained on a large data set in the future. Machine learning classifiers such as Random Forest and SVM can also be tested. As well as ResNet50 and LSTM models, deep learning models can also be used in run-time Botnet detection. Besides being integrated with front-end web applications, the research' model can also be used with back-end web applications.

## Figures and Tables

**Figure 1:** Types of Machine learning.

**Figure 2:** Flow chart for modelling.

**Figure 3:** Proposed methodology.

**Figure 4:** Attribute label plot.

**Figure 5:** Attribute “attack_cat” plot.

**Figure 6:** Attribute “state” description.

**Figure 7:** Attribute “service” description.

**Figure 8:** Skewness plots.

**Figure 9:** Pair plots of attributes “djit and dloadl”.

**Figure 10:** Attribute “ddtl” description.

**Figure 11:** Box plots of all numeric attributes.

**Figure 12:** Comparison plot of attributes “attack_cat VS no. of events”.

**Figure 13:** Pre-processing steps.

**Figure 14:** Plot of missing/null values.

**Figure 15:** Before encoding.

**Figure 16:** After encoding.

**Figure 17:** Heapmap - feature engineering.

**Figure 18:** Classification report of imbalanced data - DT.

**Figure 19:** Classification report of balanced data - DT.

**Figure 20:** Confusion matrix of imbalanced data - DT.

**Figure 21:** Classification report of balanced data - DT.

**Figure 22:** Classification report of imbalanced data - XgBoost.

**Figure 23:** Classification report of balanced data–XgBoost.

**Figure 24:** Confusion matrix of imbalanced data-XgBoost.

**Figure 25:** Confusion matrix of balanced data-XgBoost.

**Figure 26:** Classification report of imbalanced data - LR.

**Figure 27:** Classification report of balanced data - LR.

**Figure 28:** Confusion matrix of imbalanced data, LR.

**Figure 29:** Confusion matrix of balanced data, LR.

**Figure 30:** Comparative analysis of unbalanced data.

The article "Botnet Attack Detection in IoT Using Machine Learning" was published in 2022. Journal: Comput Intell Neurosci.

**Figure 31:** Comparative analysis of balanced data.

**Table 1:** Few dataset description attribute.

Sr#	Attribute	Description	DataType
**1**	Id	The unique serial number of records	Integer
**2**	Dur	Record total duration	Float
**3**	Proto	Transaction protocol	Object
**4**	Service	Http, ftp, smtp, ssh, dns, ftp-data, irc and (-) if not much used service	Object
**5**	State	Indicates to the state and its dependent protocol	Object
**6**	Spkts	Source to destination packet count	Integer
**7**	Dpkts	Destination to source packet count	Integer
**8**	Sbytes	Source to destination transaction bytes	Integer
**9**	Dbytes	Destination to source transaction bytes	Integer

**Table 2:** Accuracy table - Decision tree.

Sr#	Dataset	Train accuracy (%)	Test accuracy (%)
1	Un-balanced	100	100
2	Balanced	100	94

The classification report for both cases is.

**Table 3:** Accuracy table - XgBoost.

Sr#	Dataset	Train accuracy (%)	Test accuracy (%)
1	Imbalanced	100	100
2	Balanced	100	93

**Table 4:** Accuracy table - Logistic regression.

Sr#	Dataset	Train accuracy (%)	Test accuracy (%)
1	Unbalanced	100	100
2	Balanced	100	78

## Data Availability

The data used in this paper can be requested from the corresponding author upon request. Data will be provided on request.
